RETRACTED

# Effect Analysis of In-Hospital Transfer Care Based on STABLE Technology in Critically Ill Newborns

**DOI:** 10.1155/2022/8250655

**Published:** 2022-07-13

**Authors:** Li Fang, Jiaoru Pei, Siqiong Jiang

**Affiliations:** Department of Pediatrics, Shanghai Jiao Tong University Affiliated Six People's Hospital, Shanghai 200233, China

## Abstract

**Purpose:**

Analysis of the effectiveness of in-hospital transfer care based on the STABLE (sugar and safe care, temperature, airway, blood pressure, lab work, emotional support) technique in critically ill neonates.

**Methods:**

Retrospective analysis of the case data of 180 critically ill neonates transferred to the NICU (neonatal intensive care unit) via the delivery room (operating room) in our hospital from April 2020 to December 2021. Of which, 88 newborns from April 2020 to February 2021 were resuscitated by conventional resuscitation and then transferred to the NICU by the nurses in the delivery room (operating room) through the green channel, and they were recorded as the control group; and 92 newborns from March to December 2021 were transferred to the NICU by the NICU transfer nurses who arrived at the delivery room (operating room) earlier and used the in-hospital transfer care based on STABLE technology, and they were recorded as the intervention group. The indicators to be assessed were the execution pass rate in the simulated assessment of the transfer emergency procedure for both groups of transporters, execution times of the various subprocesses during the transfer procedure for both groups of transporters, accidents in transit, and blood glucose, blood pressure, body temperature, respiration, blood gas indicators, and family satisfaction of children in both groups after transfer.

**Results:**

The total execution pass rate for transporters was higher in the intervention group than in the control group (*P* < 0.05). The execution times of the various subprocesses during the transfer procedure of transporters were shorter in the intervention group than in the control group (*P* < 0.05). The incidence of accidents in transit was lower in the intervention group than in the control group (*P* < 0.05). After transfer, the blood glucose, blood pressure, body temperature, respiratory, and blood gas indicators of the children in the intervention group were all more stable than those in the control group (*P* < 0.05). The satisfaction of the families of the children in the intervention group was higher than that of the control group (*P* < 0.05).

**Conclusion:**

The implementation of transfer care based on STABLE technology for newborns in urgent need of in-hospital transfer can effectively improve the comprehensive quality and emergency response ability of transfer nurses and shorten the in-hospital transfer time, and the incidence of adverse reactions during the transfer of children is less, the vital signs are stable, and the satisfaction of family members is high, which is of promotion value.

RETRACTED

## 1. Introduction

About 20 million newborns are born in China every year, and 10%∼20% of them are high-risk newborns [1, 2]. These high-risk newborns have a rapid onset, rapid progression, severe illness, and high mortality rate. Due to uneven medical standards across regions, some of these high-risk newborns are at risk of death because they do not have timely access to quality medical resources. In 2009, the Neonatology Group of the Paediatrics Branch of the Chinese Medical Association conducted an epidemiological survey of neonatal deaths in 80 hospitals in 22 provinces and autonomous regions across China. The results showed that 46.4% of neonatal deaths occurred within 24 hours of hospitalisation [3] and that many of these deaths were caused by the lack of standardised resuscitation and timely referral after birth.

Neonatal transport (NT) is an important part of the work of the newborn care centre (NCC). The purpose is to safely transfer high-risk newborns to the neonatal intensive care unit (NICU) of NCC for treatment and give full play to the role of high-quality health resources [4]. However, there may be a risk of disease change and death during transport. In 1996, a neonatal education program called STABLE was implemented in the United States and by the end of 2011 had provided evidence-based education on postneonatal resuscitation and pretransport stabilisation care to more than 250,000 perinatal health team members from around the world [5]. STABLE represents six assessment parameters, namely S (sugar and safe care) to maintain stable blood glucose and safe care; T (temperature) to maintain stable body temperature; A (airway) to ensure a clear airway; B (blood pressure) to maintain stable blood pressure; L (lab work) for basic laboratory; and E (emotional support) to provide emotional support [6, 7]. The STABLE technique has been widely accepted and used in many countries and has been shown to be effective in reducing the incidence of death and maintaining normal body temperature during the transfer of high-risk newborns [8, 9]. In recent years, the STABLE technique has been increasingly applied to the out-of-hospital transfer of critically ill neonates in China, but no studies on the application of the STABLE technique to the in-hospital transfer of critically ill neonates have been reported in China. Based on the disciplinary strengths of a tertiary general hospital, this study was guided by the Guidelines for Neonatal Transport (2017 edition) [10] and established a high-risk neonatal transport team in the hospital, equipped with professional transport equipment and medications, developed a complete scheduling, handover, and training system, and provided care for high-risk neonates meeting the indications for transport according to the STABLE technique, with remarkable results. The summary is as follows.

RETRACTED

## 2. Materials and Methods

### 2.1. General Data

This study includes a retrospective analysis of the case data of 180 critically ill neonates transferred to the NICU via the delivery room (operating room) in our hospital from April 2020 to December 2021. Of which, 88 newborns from April 2020 to February 2021 were resuscitated by conventional resuscitation and then transferred to the NICU by the nurses in the delivery room (operating room) through the green channel and were recorded as the control group; and 92 newborns from March to December 2021 were transferred to the NICU by the NICU transfer nurses who arrived at the delivery room (operating room) earlier and used the in-hospital transfer care based on STABLE technology, and they were recorded as the intervention group. The comparison of baseline data in Table 1 for both groups was not significantly different and was comparable (*P* > 0.05).

### 2.2. Transfer Staff

Two transfer nurses from the NICU joined the neonatal in-hospital safe transfer care team, which also included 9 neonatologists, 8 midwives, and 10 obstetricians, making a total of 29 people.

### 2.3. High-Risk Neonatal Diagnostic Criteria

(1) Birth weight <1500 g or gestational week <32 weeks; (2) severe birth asphyxia, which remains in a critical condition after resuscitation; (3) severe respiratory distress, frequent apnoea requiring assisted ventilation; (4) cyanosis after birth that does not improve with oxygen therapy, shock, or congenital heart disease; (5) congenital anomalies requiring immediate surgical treatment; and (6) severe infection, abnormal neurobehaviour, frequent convulsions, severe jaundice requiring blood exchange, acute anaemia, frequent vomiting, diarrhoea, dehydration, etc.

### 2.4. Neonatal Inclusion Criteria

(1) Meeting the diagnostic criteria for high-risk neonates; (2) complete maternal data; and (3) informed consent of the child's family.

### 2.5. Neonatal Exclusion Criteria

(1) Those who could not be treated in our NICU and needed to be transferred to an outside hospital; (2) those who were stabilised and transferred directly to an obstetric ward; and (3) those who had died or abandoned treatment.

### 2.6. Intervention Methods

(1) Control group: resuscitated by conventional resuscitation and then transferred to the NICU from the green channel by the nurses in the delivery room (operating room). The routine transfer care process for critically ill newborns is detailed in Figure 1. (2) Intervention group: transferred to the NICU by the NICU transfer nurses who arrived at the delivery room (operating room) earlier and used the in-hospital transfer care based on STABLE technology. The key operational processes of the safe transfer care team were as follows: ① the delivery room (operating room) was kept in contact with the neonatal in-hospital transfer care team (NICU extension 58316); ② NICU nurses should familiarise themselves with the child's antenatal and intrapartum conditions, consultation and treatment, and pregnancy risk factors as soon as possible and arrived at the delivery room (operating theatre) before the foetus was delivered, communicated actively with the midwife and paediatrician, and prepared for pretransfer emergencies; ③ NICU nurses played an active role in a safe transfer care intervention based on the STABLE ambulance technique. A rapid and comprehensive assessment of the child with the paediatrician after birth was carried out, accompanied by a transfer care model based on STABLE technology to stabilise the child's condition. The details and transfer measures of STABLE technology are shown in Table 2; and ④ once the neonate was stable, the NICU transfer nurse, together with the paediatrician, would transfer the neonate directly to the NICU by the green channel in a rapid and safe manner.

RETRACTED

### 2.7. Assessment Indicators

(1) Comparison of execution pass rate in the simulated assessment of the transfer emergency procedure for both groups of transporters. The assessment consisted of four parts: item preparation (10 scores), operational processes (50 scores), operational techniques (20 scores), and effectiveness evaluation (20 scores). The total score was 100, with 80 being a pass. Trainees with a score of 95 or more could be officially admitted to the transit team shifts. (2) Comparison of execution times of the various subprocesses during the transfer procedure for both groups of transporters, including nurse arrival time (day/night), time to establish airway, time to oxygen inhalation, time to establish intravenous access, time to keep warm and shockproof, time to cardiac monitoring, and time to establish medical records. (3) Record the occurrence of accidents in transit for both groups of children. (4) Record the blood glucose, blood pressure, body temperature, and respiration of the children in both groups after the transfer. (5) Record the blood gas indicators including pH, PaO_2_, and PaCO_2_ of the children in both groups after the transfer. (6) Comparison of family satisfaction after transfer of children in both groups. A questionnaire was administered to the families of the children being transferred through a self-designed satisfaction assessment form. The questionnaire consisted of 3 aspects of transfer process (40 points), transfer technique (30 points), and service attitude (30 points) with 5 levels: very satisfied (100–90 points), satisfied (89–80 points), basically satisfied (79–60 points), dissatisfied (59–50 points), and very dissatisfied (49–0 points).

RETRACTED

### 2.8. Statistical Methods

The SPSS 21.0 statistical package was used for data analysis. The measurement data were described by $\bar{x}$ ± *s*, and ANOVA was used for comparison between groups; the count data were described by frequency and percentage, and the *χ*^2^ test was used between groups; and differences were considered statistically significant at *P* < 0.05.

## 3. Results

### 3.1. Comparison of Execution Pass Rate in the Simulated Assessment of the Transfer Emergency Procedure for Both Groups of Transporters

The total execution pass rate for transporters was higher in the intervention group than in the control group (*P* < 0.05) (Figure 2).

### 3.2. Comparison of Execution times of the Various Subprocesses during the Transfer Procedure for Both Groups of Transporters

The execution times of the various subprocesses during the transfer procedure of transporters were shorter in the intervention group than in the control group (*P* < 0.05) (Figure 3).

### 3.3. Comparison of Incidence of Accidents in Transit for Both Groups of Children

The incidence of accidents in transit was lower in the intervention group than in the control group (*P* < 0.05) (Figure 4).

### 3.4. Comparison of Blood Glucose, Blood Pressure, Body Temperature, and Respiratory for Both Groups of Children

After transfer, the blood glucose, blood pressure, body temperature, and respiratory of the children in the intervention group were all more stable than those in the control group (*P* < 0.05) (Figure 5).

### 3.5. Comparison of Blood Gas Parameters after Transfer for Both Groups of Children

After transfer, the pH, PaO_2_, and PaCO_2_ of the children in the intervention group were all more stable than those in the control group (*P* < 0.05) (Figure 6).

### 3.6. Comparison of Family Satisfaction after Transfer of Children in Both Groups

After transfer, the satisfaction of the families of the children in the intervention group was higher than that of the control group (*P* < 0.05) (Figure 7).

## 4. Discussion

Critical neonatal transport is not just a simple transport process, it is a complete emergency and monitoring system that can largely reduce neonatal morbidity and mortality and is a breakthrough in neonatal emergency technology [11]. In a study involving 346 neonatal transfers, adverse events occurred in 36% of neonates, of which 67% were human error, 21% were equipment failure, and 9% were ambulance problems [12]. To achieve safe and rapid transport, we must standardise and optimise the transport work in order to reduce complications and neonatal mortality. The purpose of traditional transport is to safely and quickly transfer critically ill neonates from primary hospitals with inadequate specialist emergency medical equipment and a lack of specialist technicians to tertiary hospital neonatal units for effective treatment and care [13, 14]. Based on the discipline advantages of the tertiary general hospital of our hospital, this study took the lead in putting forward the concept of “moving the work of NICU nurses forward.” That is, a specialist NICU nurse enters the delivery room/operating room in advance and maintains the stability of the vital signs of the critically ill newborn throughout the in-hospital transfer through STABLE transfer care by a specialist nursing team in the first instance.

RETRACTED

Improving the comprehensive quality of emergency care for transporters during transport is an important prerequisite for ensuring the quality of care for critically ill neonates [15, 16]. The transfer of critically ill newborns is different from the general transfer of children, which requires the transfer nurses to have good psychological quality, superb puncture techniques, skilled neonatal resuscitation and first aid, as well as meticulous and keen observation ability, sensitive resuscitation awareness, and good resilience [17, 18]. In contrast, the routine transportation nursing mainly includes keeping warm, keeping the respiratory tract smooth, keeping the venous channel smooth, and maintaining the stability of vital signs, and the children have not received all-round nursing in the transportation. In this result, the total execution pass rate for transporters was higher in the intervention group than in the control group. Reasons for poor emergency response by nurses include unfamiliarity with the environment, unfamiliarity with systems and work processes, inadequate skills, confusion in rescue procedures when resuscitating children, lack of clinical experience, incomplete or incorrect nursing records, and so on [19]. The implementation of the transfer protocol based on the STABLE technique in this study has made it easier for the transporters to grasp and strengthen their memory by making the entire transfer process more procedural and specific, reducing the tension and confusion of the transporters when facing an unfamiliar environment, achieving stability, accuracy, speed, and care and providing favourable conditions for the timely treatment of critically ill newborns.

RETRACTED

The transfer care based on the STABLE technique enhances the awareness and skills of the transfer staff and improves their overall coordination and resilience. Figure 3 shows that the transfer nurses in the intervention group took significantly less time to get in place (day/night), establish an airway, administer oxygen, establish intravenous access, keep warm and shockproof, perform cardiac monitoring, and establish a medical record than those in the control group. This objectively reflects that the overall emergency response capability and efficiency of the nurses have been significantly improved and that they have been able to coordinate more effectively with the doctors and other staff during the actual transport and rescue, which can win time for the rescue of critically ill children.

The crippled physiological system leaves the child without the ability to adapt to life outside the womb. Any fluctuation in blood glucose, blood pressure, or body temperature can pose a great threat to the life of the newborn, making the success of the transfer much lower or even fatal, so it is important to provide safe care for the child at all times and in all places to ensure the stability of the child's physiological system and behaviour [20, 21]. In this study, the incidence of accidents during the transfer was lower in the intervention group than in the control group; after the transfer, the blood glucose, blood pressure, body temperature, and respiratory of the children in the intervention group were all more stable than those in the control group. This may be because in-hospital transfer care based on STABLE technology not only allows the child to receive care equivalent to that of a mobile NICU, but, in the STABLE transfer model, the transfer of a critically ill newborn becomes an anticipatory and active transfer and a continuous process of monitoring and treatment, where the child's vital signs are known and life support is given, while at the same time the possible future sequelae of the baby are taken into account and proactive measures are taken to prevent them at the start of the transfer. The use of STABLE technology in the intrahospital transfer of critically ill newborns is a powerful way to improve the safety of the child and to keep the child's vital signs stable.

The results also show that in-hospital transfer care based on STABLE technology increases the satisfaction of the child's family. During the transfer of a critically ill neonate, the speed and quality of the transfer are crucial to the life and prognosis of the child. The implementation of the STABLE technique for in-hospital transfer care has transformed the previous “master-slave” relationship into a “side-by-side and complementary” partnership. As a result, team spirit has increased significantly and all members involved in the transfer process are able to perform the treatment with skill and confidence. This, together with the emotional support and assistance provided by the transport staff to the family and the encouragement of the family to face the crisis in a positive manner, resulted in a significant increase in the satisfaction of the family with the transport process.

RETRACTED

To sum up, the implementation of transfer care based on STABLE technology for newborns in urgent need of in-hospital transfer can effectively improve the comprehensive quality and emergency response ability of transfer nurses and shorten the in-hospital transfer time, and the incidence of adverse reactions during the transfer of children is less, the vital signs are stable, and the satisfaction of family members is high, which is of promotion value.

## Figures and Tables

**Figure 1:** Flowchart of routine transfer care for critically ill newborns.

**Figure 2:** Comparison of execution pass rate in the simulated assessment of the transfer emergency procedure for both groups of transporters. Note: comparison with the intervention group, ^*∗*^*P* < 0.05.

**Figure 3:** Comparison of execution times of the various subprocesses during the transfer procedure for both groups of transporters. Note: comparison with the intervention group, ^*∗*^*P* < 0.05.

**Figure 4:** Comparison of incidence of accidents in transit for both groups of children. Note: comparison with the intervention group, ^*∗*^*P* < 0.05.

**Figure 5:** Comparison of blood glucose, blood pressure, body temperature, and respiratory for both groups of children. Note: comparison with the intervention group, ^*∗*^*P* < 0.05.

**Figure 6:** Comparison of blood gas parameters after transfer for both groups of children. Note: comparison with the intervention group, ^*∗*^*P* < 0.05.

**Figure 7:** Comparison of family satisfaction after transfer of children in both groups. Note: comparison with the intervention group, ^*∗*^*P* < 0.05.

**Table 1:** Baseline data for both groups.

Items	Intervention group (*n* = 92)	Control group (*n* = 88)	*χ* ^2^/*t*	*P*
Boy/girl	49/43	47/41	0.001	0.984
Transfer of diseases/cases			1.918	0.751
Premature birth and related complications	30	29		
Neonatal asphyxia and related complications	19	21		
Respiratory abnormalities	25	20		
Digestive abnormalities	12	15		
Others	6	3		
Gestational age/weeks	37.59 ± 2.24	37.58 ± 2.09	0.031	0.975
Body weight/kg	2.82 ± 0.46	2.81 ± 0.46	0.146	0.884

RETRACTED

**Table 2:** STABLE technology specifics and transfer measures.

Factors	Transfer measures
S (sugar and safe care)	1. Assess for risk factors for hypoglycaemia: e.g., prematurity, less than gestational age, greater than gestational age, diabetic mother, stress (especially history of perinatal stress), respiratory distress, asphyxia, shock, hypothermia, sepsis, etc. 2. Target blood glucose monitoring: blood was collected from the child's heel and monitored by a rapid blood glucose meter, ensure that the child's blood glucose was maintained at 2.6–7.0 mmol/L. 3. Individual assessment according to the week of pregnancy and the cause of the hypoglycaemia. 4. The critically ill newborn shall be fasted temporarily, the venous access shall be opened, and glucose intravenous drip shall be performed according to the doctor's advice when necessary, and the drip rate shall be adjusted according to blood glucose. During infusion, monitor blood glucose every 15–30 minutes, and closely observe and keep the venous channel unblocked during infusion.

T (temperature)	1. Assess for risk factors for hypothermia: e.g., prematurity, small for gestational age, hypoxia, prolonged resuscitation, co-infections, cardiac, neurological, and endocrine problems, neonates with hypotonia, etc. 2. Target body temperature: try to maintain the body temperature at 36.5–37.2°C. 3. The temperature of delivery room (emergency room) shall be increased to 25–28°C (recommended by the World Health Organization). And preheat the warm box. 4. All articles contacting the body shall be preheated first, the wet towel shall be removed in time, and the baby shall wear a hat; <1500 g premature infants are wrapped in polyethylene (food grade plastic) from chin to foot. 5. Keep warm during all operations and rescue. Reduce the shielding of far-infrared radiation heater during rescue to ensure the good function of temperature sensor. 6. The warming box shall be used for rewarming of hypothermia newborns, and the rewarming speed shall not exceed 0.5°C per hour. 7. Transfer of critically ill and/or premature babies by preheated warming boxes.

A (airway)	1. Ensure a clear airway and remove secretions from the respiratory tract. 2. Assessment of respiration: respiratory rate and work done, shortness of breath (>60 breaths/min), aspiration concavity, distress, moaning, apnoea, pneumothorax, and assessment of heart rate and oxygen saturation. Administer oxygen as required and specify the concentration of inhaled oxygen and the method of administration. Oxygen saturation needs to be measured before and after the catheter and adjusted carefully to maintain oxygen saturation at 88%–95%. Assisted tracheal intubation with clear pre- and postintubation assistant roles and tasks to maintain effective ventilation, effective fixation of the tracheal tube, and placement of a gastric tube. 3. The insertion depth of sputum suction tube shall be determined by measurement method. It shall not be inserted too deep. The action during sputum suction shall be gentle and accurate. In case of vomiting and severe gastroesophageal reflux, indwelling a gastric tube to extract the contents of the stomach, and place in left lying position. 4. Assist with X-rays and early administration of PS (pulmonary surface active substance) for premature babies in respiratory distress as prescribed by the doctor and take care of them.

B (blood pressure)	1. Assess the cause of shock: e.g., hypovolemic, cardiogenic, and infectious. 2. Connect a cardiac monitor to monitor blood pressure, heart rate, and oxygen saturation. 3. Follow medical advice for volume expansion and pressure boosting. 4. Master the indications, configuration methods, and safe use principles of dopamine.

L (lab work)	1. Learn about the tests that need to be done after resuscitation and before transfer of the newborn, and the various laboratory indicators. Routine 4B tests include blood count, blood culture, blood glucose, blood gases. 2. Correctly collect arterial samples to understand and evaluate blood gas, oxygenation, and acid-base balance.

E (emotional support)	1. Make the family members of newborns aware of the need for newborns to be transferred to the NICU ward and the crisis they experience. 2. Provide support for newborn parents. 3. Neonatal paediatric nurse introduce families to ways in which parent-child communication can be facilitated in the NICU.

RETRACTED

## Data Availability

The primary data to support the results of this study are available at reasonable request to the corresponding author.

## References

[1] Deng Y. H., Sun Y. L., Gao D. (2016). Study on the effect of integrated management model on the follow-up effect of high-risk children. *China Maternal and Child Health Care*.

[2] Li L., Zhao H. (2016). Exploration and effectiveness of a graded management model for high-risk neonates. *Chinese Journal of Maternal and Child Health*.

[3] Neonatology Group of the Pediatrics Branch of the Chinese Medical Association (2009). Epidemiological survey of hospitalized neonates in China. *Chinese Journal of Contemporary Pediatrics*.

[4] Goswami I., Redpath S., Langlois R. G., Green J. R., Lee K. S., Whyte H. E. A. (2020). Whole-body vibration in neonatal transport: a review of current knowledge and future research challenges. *Early Human Development*.

[5] Kendall A. B., Scott P. A., Karlsen K. A. (2012). The S.T.A.B.L.E® Program: the evidence behind the 2012 update. *Journal of Perinatal and Neonatal Nursing*.

[6] Taylor R. M., Price-Douglas W. (2008). The S.T.A.B.L.E. Program: postresuscitation/pretransport stabilization care of sick infants. *Journal of Perinatal and Neonatal Nursing*.

[7] O’Neill N., Howlett A. A. (2007). Evaluation of the impact of the S.T.A.B.L.E. Program on the pretransport care of the neonate. *Neonatal Network*.

[8] Mathews T. J., MacDorman M. F. (2012). Infant mortality statistics from the 2008 period linked birth/infant death data set. *National Vital Statistics Reports*.

[9] Diehl-Svrjcek B. C., Price-Douglas W., Flagg J. (2011). Neonatal glucose testing via prompted intervention during the pretransport phase of care. *Advances in Neonatal Care*.

[10] Chinese Physicians Association Neonatal Specialty Committee (2017). Guidelines for neonatal transport in China (2017 edition). *Electronic Journal of Developmental Medicine*.

[11] Aagaard H., Hall E. O. C., Ludvigsen M. S., Uhrenfeldt L., Fegran L. (2018). Parents’ experiences of neonatal transfer. A meta-study of qualitative research 2000–2017. *Nursing Inquiry*.

[12] Lim M. T. C., Ratnavel N. (2008). A prospective review of adverse events during interhospital transfers of neonates by a dedicated neonatal transfer service. *Pediatric Critical Care Medicine*.

[13] Kunz S. N., Dukhovny D., Profit J., Mao W., Miedema D., Zupancic J. A. F. (2019). Predicting successful neonatal retro-transfer to a lower level of care. *The Journal of Pediatrics*.

[14] Trevisanuto D., Cavallin F., Loddo C. (2021). Trends in neonatal emergency transport in the last two decades. *European Journal of Pediatrics*.

[15] Baleine J. F., Fournier-Favre P., Fabre A. (2016). Neonatal transport characteristics. *Soins—Pediatrie, Puericulture*.

[16] Moreno Hernando J., Thió Lluch M., Salguero García E. (2013). Recommendations for neonatal transport. *Anales de Pediatría*.

[17] (2019). Group of pediatric disaster, pediatric society, Chinese medical association; pediatrics committee, medical association of Chinese People’s liberation army. *Zhong Guo Dang Dai Er Ke Za Zhi*.

[18] Liu J., Li Z., Zhang Q. (2018). Challenges in the pain assessment during neonatal transport: an update. *Minerva Pediatrica*.

[19] Pai V. V., Kan P., Gould J. B., Hackel A., Lee H. C. (2020). Clinical deterioration during neonatal transport in California. *Journal of Perinatology*.

[20] Kawaguchi A., Gunz A., de Caen A. (2019). Cross-sectional survey of Canadian pediatric critical care transport. *Pediatric Emergency Care*.

RETRACTED

[21] Zhang X. F., Li Y., Xiao G. H. (2012). Application of regionalized critical neonatal emergency transport system. *Zhong Guo Dang Dai Er Ke Za Zhi*.

